The article "Minimally Invasive Approaches for High-Risk and Elderly Patients With Acute Cholecystitis: A Systematic Review of Techniques and Outcomes" was retracted in 2025. Reasons: unreliable results or conclusions; concerns about the authorship.

# Minimally Invasive Approaches for High-Risk and Elderly Patients With Acute Cholecystitis: A Systematic Review of Techniques and Outcomes

**DOI:** 10.7759/cureus.78271

**Published:** 2025-01-30

**Authors:** Mark Abdelmaseeh, Asem Mhmndar, Ayesha Siddiqa, Shoaib S Ahamed, Kanwal Sheraz, Ahmad F Mohd, Haider Ali, Abdullah Shehryar, Abdur Rehman, Khakan Murtaza

**Affiliations:** 1 General Surgery, Assiut University, Assiut, EGY; 2 Internal Medicine, Thumbay University Hospital, Ajman, ARE; 3 Internal Medicine, Rehman Medical Institute, Peshawar, PAK; 4 Gastroenterology, Nottingham University Hospitals NHS Trust, Nottingham, GBR; 5 General Surgery, Mayo Hospital, Lahore, PAK; 6 Internal Medicine, Allama Iqbal Medical College, Lahore, PAK; 7 Surgery, Mayo Hospital, Lahore, PAK; 8 Internal Medicine, Nishtar Medical University, Multan, PAK

**Keywords:** acute cholecystitis, elderly patients, high-risk patients, laparoscopic cholecystectomy, minimally invasive surgery, patient-centered care, percutaneous cholecystostomy, postoperative drainage, randomized controlled trials

## Abstract

Acute cholecystitis is a prevalent condition marked by gallbladder inflammation, typically due to gallstone obstruction, and poses management challenges, particularly for high-risk and elderly patients. This systematic review compares the efficacy and safety of two minimally invasive approaches: percutaneous drainage methods, such as percutaneous cholecystostomy, and laparoscopic cholecystectomy (LC). A structured search of PubMed, MEDLINE, and Embase was conducted, yielding six randomized controlled trials that met the inclusion criteria. Findings suggest that percutaneous drainage combined with LC offers advantages in reducing operative time, hospital stay, and complication rates, particularly for high-risk patients, compared to LC alone. However, routine postoperative drainage after LC may contribute to prolonged hospital stays and increased postoperative pain without reducing morbidity. Advanced energy devices, such as harmonic scalpels, may further optimize surgical outcomes, though benefits are limited. This review highlights the importance of patient-centered, selective approaches over routine practices, advocating for personalized strategies that prioritize patient safety and recovery. Future research should refine patient selection criteria and evaluate long-term outcomes to establish more precise guidelines for managing acute cholecystitis in vulnerable populations.

## Introduction and background

Acute cholecystitis, an inflammation of the gallbladder typically caused by gallstone obstruction, remains a common yet challenging condition to manage, particularly in high-risk or elderly patients [1]. Traditionally, treatment has focused on emergency surgery or drainage techniques to mitigate inflammation, alleviate symptoms, and prevent complications such as gallbladder perforation. However, there is an ongoing debate regarding the optimal management approach, especially when considering minimally invasive procedures [2]. Advances in laparoscopic techniques have allowed for safer and more effective surgical interventions, such as laparoscopic cholecystectomy (LC), which has become a gold standard for treating gallstone-related cholecystitis [3]. Nevertheless, percutaneous drainage methods, including percutaneous cholecystostomy, offer a less invasive alternative, especially for patients who may not be ideal surgical candidates.

The article "Minimally Invasive Approaches for High-Risk and Elderly Patients With Acute Cholecystitis: A Systematic Review of Techniques and Outcomes" was retracted in 2025. Reasons: unreliable results or conclusions; concerns about the authorship.

Minimally invasive approaches, such as LC and percutaneous drainage, are increasingly utilized to balance treatment efficacy with patient safety [4]. According to the Revised Tokyo Guidelines (TG18), percutaneous drainage, particularly percutaneous cholecystostomy, is recommended in patients with Grade III (severe) acute cholecystitis or those deemed unfit for immediate surgery due to high surgical risks. LC, the gold standard for gallbladder removal, aims to definitively address the underlying pathology and prevent recurrence, whereas drainage techniques are designed to provide temporary symptom relief and infection control [5]. Despite the clarity provided by these guidelines, the comparative efficacy, safety, and outcomes associated with these approaches remain subjects of an ongoing debate. While evidence suggests that elderly and high-risk patients benefit more from drainage due to its reduced surgical risks, timely cholecystectomy remains critical for preventing recurrent inflammation and complications [6]. This systematic review consolidates evidence from recent studies to better define the role of these minimally invasive approaches in managing acute cholecystitis, particularly within the context of guideline recommendations.

This systematic review evaluates various minimally invasive approaches for managing acute cholecystitis in elderly and high-risk patients. The study applies a modified PICO framework [7] to guide the synthesis of evidence. The Population includes adult patients diagnosed with acute cholecystitis, with particular attention to elderly and high-risk individuals. The Interventions encompass a range of minimally invasive techniques, including percutaneous drainage (e.g., percutaneous cholecystostomy), LC, the use of harmonic scalpels versus monopolar electrosurgical energy, and postoperative drainage strategies (routine vs. selective). The Comparisons include alternative minimally invasive methods, such as LC alone or the omission of routine drainage. The Outcomes of interest include safety, efficacy, operative time, complication rates, hospital stays, postoperative pain, and long-term recovery. By evaluating different minimally invasive strategies, this review aims to provide a comprehensive understanding of their relative benefits and limitations, guiding clinicians in tailoring approaches to the needs of vulnerable patient populations.

The article "Minimally Invasive Approaches for High-Risk and Elderly Patients With Acute Cholecystitis: A Systematic Review of Techniques and Outcomes" was retracted in 2025. Reasons: unreliable results or conclusions; concerns about the authorship.

## Review

Materials and methods

Search Strategy

The search strategy for this systematic review was designed to capture comprehensive and relevant studies comparing minimally invasive approaches, such as percutaneous drainage and LC, in the management of acute cholecystitis, particularly among high-risk and elderly patients. Databases including PubMed, MEDLINE, and Embase were systematically searched using key terms and medical subject headings (MeSH), such as “acute cholecystitis,” “percutaneous cholecystostomy,” “laparoscopic cholecystectomy,” and “postoperative drainage.” Additional terms like “high-risk patients,” “ultrasonic energy,” and “hospital stay” were used to refine the results and ensure the inclusion of studies relevant to this patient population. Only randomized controlled trials (RCTs) published in English were included, focusing on studies conducted within the last two decades to ensure the latest surgical advancements were represented. The search strategy adhered to PRISMA (Preferred Reporting Items for Systematic Reviews and Meta-Analyses) guidelines [8], ensuring a transparent and replicable approach to study selection, screening, and data extraction. This structured search and adherence to the PRISMA methodology strengthened the review’s comprehensiveness and relevance.

Eligibility Criteria

The eligibility criteria for this systematic review were carefully defined to ensure that only high-quality, relevant studies were included. Eligible studies were RCTs published in English, as these provide the most rigorous evidence for comparing minimally invasive approaches in managing acute cholecystitis. Studies needed to focus specifically on high-risk or elderly patients with acute cholecystitis, comparing percutaneous cholecystostomy (PC), ultrasound-guided percutaneous drainage, or similar drainage techniques with LC or assessing the impact of postoperative drainage versus no drainage. Studies were excluded if they involved non-randomized designs, observational studies, or lacked comparative data on the specified interventions. Additionally, trials focusing on patients with non-acute cholecystitis, pediatric populations, or those addressing alternative surgical or non-surgical treatments were excluded to maintain a clear focus on the target patient group and interventions. Only studies published within the last two decades were included to capture recent advancements in minimally invasive surgical techniques, ensuring the findings remain relevant to current clinical practice.

The article "Minimally Invasive Approaches for High-Risk and Elderly Patients With Acute Cholecystitis: A Systematic Review of Techniques and Outcomes" was retracted in 2025. Reasons: unreliable results or conclusions; concerns about the authorship.

Data Extraction

The data extraction process for this review focused on systematically gathering essential information from each eligible RCT on minimally invasive approaches for managing acute cholecystitis in high-risk and elderly patients. For each study, we extracted data on patient demographics (age, comorbidities, risk level), intervention details (e.g., PC, ultrasound-guided drainage, or LC), and specific drainage protocols when applicable. Key outcomes included operative duration, hospital stay length, complication rates, conversion rates to open surgery, and mortality. Secondary outcomes, such as postoperative pain scores and cost considerations, were also collected. Statistical data, including p-values and confidence intervals, were recorded to assess the significance of findings. This structured approach, aligned with PRISMA guidelines, facilitated a thorough synthesis of data to compare the efficacy and safety of each intervention in this patient population.

Data Analysis and Synthesis

The data analysis and synthesis for this review involved a comparative approach to evaluate the efficacy and safety of minimally invasive interventions, specifically percutaneous drainage techniques and LC, in high-risk and elderly patients with acute cholecystitis. Quantitative data, including operative times, hospital stays, complication rates, and postoperative pain scores, were reviewed and compared across studies to identify trends in outcomes between interventions. Descriptive synthesis was employed to examine secondary outcomes, such as cost-effectiveness and procedural feasibility, due to variability in reporting among studies. Statistical significance was noted where reported, with particular focus on clinically relevant findings such as reductions in operative duration and complication rates. This approach allowed for a cohesive synthesis of evidence, highlighting both the benefits and limitations of each intervention and providing insights into optimal management strategies for this high-risk patient group.

Results

Study Selection Process

The study selection process for this systematic review followed a structured approach, adhering to PRISMA guidelines to ensure transparency and rigor. A total of 319 records were initially identified across three databases: PubMed (120), MEDLINE (105), and Embase (94). After removing 88 duplicate records, 231 unique studies were screened for relevance based on titles and abstracts. Of these, 101 studies were excluded, leaving 130 reports for further retrieval. However, 86 reports could not be retrieved, resulting in 44 studies that were fully assessed for eligibility. During this eligibility assessment, 38 studies were excluded due to non-RCT designs (15), lack of focus on high-risk or elderly patients (10), absence of comparative data on specified interventions (8), and focus on pediatric or non-acute cholecystitis populations (5). Ultimately, six studies met all eligibility criteria and were included in the final review. This systematic selection process ensured that only relevant, high-quality studies were incorporated into the analysis. Figure 1 represents the study selection process.

The article "Minimally Invasive Approaches for High-Risk and Elderly Patients With Acute Cholecystitis: A Systematic Review of Techniques and Outcomes" was retracted in 2025. Reasons: unreliable results or conclusions; concerns about the authorship.

**Figure 1:** The PRISMA flowchart represents the study selection process. PRISMA: Preferred Reporting Items for Systematic Reviews and Meta-Analyses; RCT: Randomized Controlled Trial

Characteristics of the Selected Studies

The selected studies in this review encompass a range of RCTs focused on evaluating minimally invasive approaches in managing acute cholecystitis, particularly in high-risk and elderly patients. Each study involved a distinct intervention and comparison group, such as percutaneous drainage techniques combined with LC versus LC alone, or the use of ultrasonic energy versus monopolar electrosurgical energy in LC. Outcomes commonly assessed across these studies included operative time, hospital stay length, complication rates, postoperative pain, and cost-effectiveness. Collectively, the studies provide insights into the efficacy and safety of various techniques, with findings that support the potential benefits of staged and selective approaches in reducing operative time, recovery period, and associated complications in high-risk patient populations. Table 1 details the study characteristics, interventions, outcomes, and key findings.

**Table 1:** Summary of the key randomized controlled trials comparing minimally invasive approaches for managing acute cholecystitis. PTGD: Percutaneous Transhepatic Gallbladder Drainage; LC: Laparoscopic Cholecystectomy; AIGB: Acutely Inflamed Gallbladder; APACHE-II: Acute Physiology and Chronic Health Evaluation II; ACC: Acute Calculous Cholecystitis; PC: Percutaneous Cholecystostomy; PCLC: Percutaneous Cholecystostomy followed by Early Laparoscopic Cholecystectomy; DLC: Delayed Laparoscopic Cholecystectomy

Authors (Year)	Study Design	Population	Age (Mean/Median)	Risk Grading	Intervention	Comparison	Outcomes	Statistical Findings	Key Findings/Conclusion
Hu et al. (2015) [9]	Randomized Controlled Trial	Seventy elderly and high-risk patients with acute cholecystitis (35 in intervention, 35 in the control group)	Mean: 75 years	High risk (based on comorbidities, surgical fitness)	B-mode ultrasound-guided percutaneous transhepatic gallbladder drainage (PTGD) combined with laparoscopic cholecystectomy (LC)	Laparoscopic cholecystectomy (LC) alone	Duration of operation, postoperative length of hospital stay, volume of bleeding, conversion rate to laparotomy, complication rate	Operation time: 55.6 ± 23.3 min vs. 91.35 ± 25.1 min; Hospital stay: 3.0 ± 1.3 days vs. 7.0 ± 1.7 days; Bleeding: 28.7 ± 15.2 ml vs. 60.38 ± 16.4 ml; Conversion: 3 vs. 10; Complications: 3 vs. 8 (all p < 0.05)	PTGD + LC significantly improved safety and efficacy in managing acute cholecystitis in elderly and high-risk patients compared to LC alone, with shorter operation time, faster recovery, and fewer complications.
Zanghì et al. (2014) [10]	Randomized Controlled Trial	One hundred and sixty-four patients undergoing laparoscopic cholecystectomy (121 in the traditional group, 43 in the harmonic scalpel group)	Median: 65 years	Moderate to low risk	Ultrasonic (harmonic) energy for dissection and closure of cystic artery and duct	Monopolar electrosurgical energy	Operative time, gallbladder perforation rate, intraoperative blood loss, postoperative drainage, hospital stay	Operative time: 35.36 ± 10.15 min vs. 55.6 ± 12.10 min (p < 0.0001); Perforation: 6.98% vs. 20.66% (p < 0.05); Blood loss: 12.41 ± 8.22 ml vs. 29.32 ± 14.21 ml (p < 0.0001); Hospital stay: 48.15 ± 4.29 h vs. 49.06 ± 2.94 h (p > 0.05)	Harmonic scalpel significantly reduced operative time, blood loss, and gallbladder perforation rate, but no difference in overall morbidity. Wider adoption is not recommended as benefits are limited.
Kim et al. (2015) [11]	Randomized Controlled Trial	One hundred and ninety-three patients with acutely inflamed gallbladder (AIGB) undergoing laparoscopic cholecystectomy	Mean: 61 years	Mild to moderate risk	Routine drain insertion after LC (Group A)	No drain insertion after LC (Group B)	Postoperative morbidities, pain levels, hospital stay, operative time	Pain at 24h: 3.9 ± 1.4 (Group A) vs. 3.3 ± 2.0 (Group B) (p = 0.014); Pain at 48h: 2.1 ± 1.5 (Group A) vs. 1.5 ± 1.4 (Group B) (p = 0.006); No significant difference in morbidity	Routine drain insertion did not reduce morbidities but increased pain and should be reconsidered in LC for AIGB.
Kortram et al. (2012) [12]	Randomized Controlled Trial (Protocol)	High-risk patients (APACHE-II score 7-14) with acute calculous cholecystitis, 284 patients across 30 hospitals	Not available	High risk (APACHE-II 7-14)	Percutaneous cholecystostomy	Laparoscopic cholecystectomy	Major complications within 3 months, re-intervention need, mortality, secondary outcomes (complications, hospital stay, procedure difficulty, total costs)	N/A (protocol publication; statistical data not available)	Designed to determine whether percutaneous cholecystostomy is superior to LC for high-risk patients; aims to establish evidence-based guidelines.
Prevot et al. (2016) [13]	Randomized Controlled Trial (Post Hoc Analysis)	Four hundred and fourteen patients with mild or moderate acute calculous cholecystitis (ACC), undergoing laparoscopic cholecystectomy	Mean: 58 years	Mild to moderate risk	Abdominal drainage post-laparoscopic cholecystectomy	No abdominal drainage	Incisional site infection (deep/superficial), distant infections, overall morbidity, readmission rate, hospital stay	Deep infection rate: 1.1% (drainage) vs. 0.8% (no drainage) (p = 0.78); Hospital stay: 5.1 days (drainage) vs. 3.3 days (no drainage) (p = 0.003)	Abdominal drainage did not improve outcomes and was associated with longer hospital stays. Routine use after LC for mild/moderate ACC may not be beneficial.
Akyürek et al. (2005) [14]	Randomized Controlled Trial	Sixty-one high-risk patients with acute calculous cholecystitis (31 in the PCLC group, 30 in the DLC group)	Mean: 73 years	High risk (based on comorbidities)	Percutaneous cholecystostomy (PC) followed by early laparoscopic cholecystectomy (LC)	Conservative treatment followed by delayed LC	Symptom relief, hospital stay, conversion rate, complication rate, cost	PC + early LC led to symptom relief within 24 hours; Early LC success rate: 93.5% (PCLC) vs. 86.6% (DLC); Shorter hospital stay and lower costs in the PCLC group	PC stabilized high-risk patients, allowing safe early LC with reduced hospital stay and cost compared to delayed LC.

Quality Assessment

Table 2 provides a detailed evaluation of six foundational studies assessing minimally invasive approaches for acute cholecystitis. The studies were appraised using standardized tools, such as the CONSORT Checklist and PRISMA Protocol Assessment, focusing on critical aspects of methodological quality. Randomization was generally adequate across studies, ensuring unbiased allocation of participants, while blinding was performed and clearly described in some cases but absent in others. Sample size justification was variable, with several studies providing it while others lacked sufficient detail. Outcome reporting was consistently clear, except for one study still at the protocol stage. Risk of bias ranged from low to moderate, with one study being unassessable due to its protocol-only status. Overall, the assessment highlights variability in study quality, with some demonstrating high methodological rigor and others identifying opportunities for improvement in future research design.

The article "Minimally Invasive Approaches for High-Risk and Elderly Patients With Acute Cholecystitis: A Systematic Review of Techniques and Outcomes" was retracted in 2025. Reasons: unreliable results or conclusions; concerns about the authorship.

**Table 2:** Quality assessment of included studies. CONSORT: Consolidated Standards of Reporting Trials; PRISMA: Preferred Reporting Items for Systematic Reviews and Meta-Analyses

Study	Tool Used	Randomization	Blinding	Sample Size Justification	Outcome Reporting	Risk of Bias	Overall Quality
Hu et al. [9]	CONSORT Checklist	Adequate	Not performed	Provided	Clear	Low	High
Zanghì et al. [10]	CONSORT Checklist	Adequate	Performed and Clear	Provided	Clear	Low to Moderate	High
Kim et al. [11]	CONSORT Checklist	Adequate	Performed and Clear	Not Mentioned	Clear	Moderate	Moderate
Kortram et al. [12]	PRISMA Protocol Assessment	Protocol Only	Protocol Only	Protocol Only	Not Reported	Not Assessable	Low
Prevot et al. [13]	CONSORT Checklist	Adequate	Not performed	Not Mentioned	Clear	Moderate	Moderate
Akyürek et al. [14]	CONSORT Checklist	Adequate	Performed and Clear	Not Mentioned	Clear	Low to Moderate	Moderate to High

Discussion

Minimally Invasive Techniques and Postoperative Drainage

This study highlights the effectiveness of minimally invasive approaches in managing acute cholecystitis, particularly in high-risk and elderly patients. Among these methods, percutaneous transhepatic gallbladder drainage (PTGD) combined with LC showed notable advantages over LC alone, as demonstrated in one included study (Hu et al. [9]). PTGD significantly reduced operative times (55.6 ± 23.3 min vs. 91.35 ± 25.1 min, p < 0.05), hospital stays (3.0 ± 1.3 days vs. 7.0 ± 1.7 days, p < 0.05), and bleeding volumes (28.7 ± 15.2 ml vs. 60.38 ± 16.4 ml, p < 0.05). Similarly, PC followed by early LC provided rapid symptom relief within 24 hours and reduced both hospital stays and treatment costs compared to delayed LC. This staged approach appears particularly beneficial for high-risk patients, allowing stabilization before definitive surgery. The use of advanced surgical tools, such as the harmonic scalpel, further enhanced outcomes during LC by decreasing operative time, blood loss, and gallbladder perforation rates compared to traditional monopolar energy. However, its impact on hospital stays and overall morbidity remained limited.

Postoperative drainage practices were also evaluated, revealing that routine drain insertion may not offer significant benefits. Instead, it was associated with increased postoperative pain at 24 hours (3.9 ± 1.4 vs. 3.3 ± 2.0, p = 0.014) and 48 hours (2.1 ± 1.5 vs. 1.5 ± 1.4, p = 0.006), as well as prolonged hospital stays in mild to moderate cases of cholecystitis (5.1 vs. 3.3 days, p = 0.003). These findings suggest that routine drainage could hinder recovery rather than improve outcomes, advocating for a more selective and patient-centered approach to postoperative care [15].

The article "Minimally Invasive Approaches for High-Risk and Elderly Patients With Acute Cholecystitis: A Systematic Review of Techniques and Outcomes" was retracted in 2025. Reasons: unreliable results or conclusions; concerns about the authorship.

PTGD is typically indicated for patients with biliary obstruction and elevated bilirubin levels caused by extrahepatic biliary outflow obstruction. However, its role extends to high-risk and elderly patients with acute cholecystitis who are unfit for immediate surgery due to significant comorbidities or hemodynamic instability. In such cases, PTGD serves as a bridge to definitive treatment by alleviating inflammation and controlling infection, thereby stabilizing the patient for safer LC. This staged approach has been shown to reduce operative times, hospital stays, and complications, as demonstrated in the study by Hu et al. [9], making it a valuable option in managing this vulnerable population.

Key Findings from RCTs

A comparative analysis of six RCTs highlights the advantages of minimally invasive strategies for managing acute cholecystitis in high-risk patients (Table 3). One included study (Hu et al. [9]) demonstrated that PTGD combined with LC was safer and more effective for high-risk patients, with reduced operative times, hospital stays, and bleeding complications compared to LC alone. The trials also revealed that the routine use of postoperative drainage may not improve patient outcomes and, in some cases, could prolong hospital stays. These findings suggest that routine drainage protocols may need to be reconsidered, especially for patients with mild to moderate cholecystitis.

**Table 3:** Comparative analysis of key outcomes from included studies. PTGD: Percutaneous Transhepatic Gallbladder Drainage; LC: Laparoscopic Cholecystectomy; PC: Percutaneous Cholecystostomy; N/A: Not Available; h: Hours

Study	Intervention	Comparison	Operative Time (min)	Hospital Stay (days)	Complication Rate	Key Conclusion
Hu et al. (2015) [9]	PTGD + LC	LC alone	55.6 vs. 91.35	3.0 vs. 7.0	3 vs. 8	PTGD + LC improves safety and efficacy in high-risk patients.
Zanghì et al. (2014) [10]	Harmonic scalpel for LC	Monopolar electrosurgical energy	35.36 vs. 55.6	48.15 h vs. 49.06 h	Lower with harmonic scalpel	Harmonic scalpel reduces operative time, blood loss, and perforation rate.
Kim et al. (2015) [11]	Routine drain insertion after LC	No drain insertion after LC	N/A	N/A	Higher in routine drain group	Routine drainage does not reduce morbidity and increases pain.
Kortram et al. (2012) [12]	Percutaneous cholecystostomy	Laparoscopic cholecystectomy	N/A	N/A	N/A	Designed to determine superiority of PC over LC in high-risk patients.
Prevot et al. (2016) [13]	Abdominal drainage post-LC	No abdominal drainage	N/A	5.1 vs. 3.3	No significant difference	Routine drainage does not improve outcomes and prolongs hospital stay.
Akyürek et al. (2005) [14]	PC + early LC	Conservative treatment + delayed LC	N/A	Lower in PC + LC	Lower in PC + LC	PC allows for symptom relief and safe early LC with reduced hospital stay.

The use of advanced energy devices, such as harmonic scalpels, further optimized surgical procedures by reducing operative time and blood loss. However, their impact on overall morbidity remains inconclusive, highlighting the need for more robust evidence on long-term outcomes. Overall, these trials underscore the importance of tailoring minimally invasive approaches to patient risk profiles, moving away from one-size-fits-all protocols toward more selective, patient-centered practices, especially in vulnerable populations.

The article "Minimally Invasive Approaches for High-Risk and Elderly Patients With Acute Cholecystitis: A Systematic Review of Techniques and Outcomes" was retracted in 2025. Reasons: unreliable results or conclusions; concerns about the authorship.

Comparative Synthesis of Key Findings

The studies highlight that percutaneous drainage methods, such as PTGD and PC, reduce operative time and hospital stays, making them safer options for high-risk patients compared to LC. However, evidence on routine postoperative drainage remains inconsistent, with some studies linking it to increased pain and delayed recovery without reducing morbidity. While advanced energy devices like harmonic scalpels improve intraoperative efficiency, their long-term impact is unclear. These findings underscore the need for stronger evidence on patient selection and drainage protocols to refine clinical guidelines and integrate emerging technologies effectively.

Alignment with Existing Literature and Drainage Controversies

This review aligns with existing literature demonstrating that PC is a viable alternative to immediate cholecystectomy in high-risk patients, providing symptom relief and reducing surgical risks. Notably, the CHOCOLATE trial reported fewer complications with LC compared to percutaneous drainage in high-risk cases, reinforcing the benefits of surgical intervention when feasible [16,17].

However, the evidence on routine postoperative drainage remains mixed. Some studies have shown that routine drains do not reduce complications but instead increase pain and prolong recovery [18,19]. The current review supports these findings, suggesting that routine drainage may delay recovery without improving outcomes. Overall, this review highlights the importance of patient-specific approaches, emphasizing minimally invasive techniques tailored to individual risk profiles to optimize outcomes [20].

Risk-Based Algorithm and Trends in Acute Cholecystitis Management

Managing acute calculous cholecystitis in high-risk patients requires a personalized approach balancing safety and clinical outcomes. This review supports a risk-based algorithm for optimizing treatment. For low to moderate-risk patients, early LC remains the gold standard, offering definitive treatment and reducing recurrence risk. In contrast, high-risk patients with significant comorbidities or elevated APACHE-II scores benefit more from percutaneous drainage followed by delayed LC, allowing initial stabilization before surgery. In critically ill patients, conservative management with antibiotics and close monitoring is preferable to minimize immediate surgical risks.

The article "Minimally Invasive Approaches for High-Risk and Elderly Patients With Acute Cholecystitis: A Systematic Review of Techniques and Outcomes" was retracted in 2025. Reasons: unreliable results or conclusions; concerns about the authorship.

Future management trends point to the integration of machine learning models and AI-driven decision support systems for risk stratification and treatment planning. These tools could enhance outcome predictions and guide intervention choices based on patient data. Additionally, advancements like robotic-assisted LC and improved imaging technologies may further reduce operative risks and recovery times. In resource-limited settings, remote monitoring and telemedicine solutions could address gaps in care delivery. Future research should refine risk prediction models and explore the long-term impact of emerging technologies to develop more precise, patient-centered guidelines. Table 4 provides a summary of the proposed algorithm and future trends.

**Table 4:** The risk-based algorithm and future trends.

Patient Risk Level	Recommended Approach	Advantages	Limitations	Future Trends
Low to Moderate Risk	Early laparoscopic cholecystectomy (LC)	Definitive treatment; reduces recurrence risk; shorter hospital stay	Potential complications in patients with unknown comorbidities	AI-driven risk prediction models to optimize patient selection
High Risk (APACHE-II > 7)	Percutaneous drainage followed by delayed LC	Allows initial stabilization; safer for patients with comorbidities	Requires follow-up surgery; may prolong overall treatment timeline	Use of robotic-assisted LC and advanced imaging modalities
Critically Ill	Conservative management with antibiotics and close monitoring	Reduces immediate surgical risk in critically ill patients	Does not address the underlying cause; risk of disease progression	Remote monitoring technologies and telemedicine consultations

Minimally Invasive Strategies and the Future of Patient-Centered Care

This review highlights that PC combined with LC significantly improves outcomes in high-risk and elderly patients with acute cholecystitis [21]. Clinically, this staged approach stabilizes patients with severe comorbidities, reducing morbidity, recovery times, and healthcare costs [22]. Additionally, the review underscores the limitations of routine postoperative drainage, which may increase pain without reducing morbidity, supporting a more selective approach tailored to patient profiles.

The article "Minimally Invasive Approaches for High-Risk and Elderly Patients With Acute Cholecystitis: A Systematic Review of Techniques and Outcomes" was retracted in 2025. Reasons: unreliable results or conclusions; concerns about the authorship.

The integration of advanced technologies, such as AI-driven risk tools and novel energy devices, can further optimize patient selection and surgical precision. In resource-limited settings, telemedicine and remote monitoring can bridge care gaps, ensuring equitable access to best practices. Revising guidelines to incorporate these innovations will help standardize patient-centered care, reduce complications, and improve long-term outcomes.

Strengths and Limitations of the Review

One of the primary strengths of this review lies in its comprehensive inclusion of multiple RCTs that assess various minimally invasive approaches, such as PC and LC, in managing acute cholecystitis in high-risk populations. The use of RCTs enhances the reliability of findings by minimizing bias and allowing for a controlled comparison of different interventions. Additionally, the focus on high-risk and elderly patients fills a gap in current literature, addressing an area of critical clinical need where traditional surgical approaches often carry high morbidity and mortality risks.

However, several limitations must be acknowledged. There is significant heterogeneity among the included studies, as each was designed with different protocols, patient populations, and intervention groups. The diversity in intervention types, such as percutaneous drainage, harmonic scalpel use, and postoperative drainage strategies, further contributes to this variability. Additionally, the relatively small sample sizes in some studies may limit the generalizability of the findings to broader populations. Variations in definitions of postoperative outcomes and drainage techniques introduce challenges in synthesizing the data, which could impact the interpretation of aggregated results. Recognizing these limitations provides a balanced perspective, emphasizing the need for further large-scale, standardized studies to better compare minimally invasive techniques and refine clinical guidelines.

Future Directions in Minimally Invasive Approaches

Future research should focus on refining patient selection criteria to improve outcomes in high-risk and elderly patients with acute cholecystitis. Advanced risk stratification tools can help identify those who would benefit most from staged interventions, such as PC followed by LC, rather than immediate surgery. Investigating long-term outcomes, including survival rates, recurrence, and quality of life, is essential to evaluate treatment efficacy comprehensively over time.

Further exploration is needed to define specific cases where postoperative drainage may aid recovery, moving away from routine use that may increase postoperative pain and delay recovery. Incorporating patient-reported outcomes, like pain levels and satisfaction, alongside clinical metrics, would better align protocols with patient-centered care goals. Technological advancements, such as AI-driven predictive models and robotic-assisted surgeries, can optimize surgical precision and reduce perioperative risks. These innovations hold particular promise in resource-limited settings, where remote monitoring tools and telemedicine consultations can bridge gaps in care. Addressing these areas in future studies will contribute to the development of evidence-based, tailored guidelines for managing acute cholecystitis more effectively and equitably [23,24].

The article "Minimally Invasive Approaches for High-Risk and Elderly Patients With Acute Cholecystitis: A Systematic Review of Techniques and Outcomes" was retracted in 2025. Reasons: unreliable results or conclusions; concerns about the authorship.

## Conclusions

This review underscores the growing importance of minimally invasive strategies in managing acute cholecystitis, particularly among high-risk and elderly patients who are less suited for immediate surgical intervention. Techniques such as PC combined with LC provide a safer, staged approach that balances the need for symptom relief with surgical risk reduction. The analysis also questions the long-standing practice of routine postoperative drainage, showing that it may increase pain and delay recovery without significantly reducing complications, advocating for a more selective, patient-specific approach. Additionally, the adoption of advanced surgical tools, such as harmonic scalpels, demonstrates the potential to optimize intraoperative efficiency, though their long-term impact requires further study. These findings align with evolving clinical trends that emphasize risk stratification and personalized care, suggesting that future guidelines should incorporate AI-driven tools and remote monitoring technologies to enhance patient selection and improve outcomes. By addressing critical gaps in the literature, this review offers actionable insights for refining surgical protocols and advancing minimally invasive techniques in both resource-rich and resource-limited settings.
